# Intervention of WeChat Group Guidance in Rapid Rehabilitation after Gynecological Laparoscopic Surgery

This article has been retracted.

**DOI:** 10.1155/2021/8914997

**Published:** 2021-09-29

**Authors:** Jing Wang, Yingying Lin, Ying Wei, Xiuying Chen, Yuping Wang, Longxin Zhang, Min Zhou

**Affiliations:** ^1^Department of Anesthesiology, Fujian Maternity and Child Health Hospital, Affiliated Hospital of Fujian Medical University, Fuzhou 350001, China; ^2^Department of Healthcare, Fujian Maternity and Child Health Hospital, Affiliated Hospital of Fujian Medical University, Fuzhou 350001, China

## Abstract

Gynecological laparoscopic surgery is the current routine treatment. Although the injury is relatively small, it is still a traumatic operation and also increases the recovery speed of patients. This paper mainly explores the intervention effect of rapid rehabilitation after gynecological laparoscopic surgery by means of WeChat group guidance based on the information adoption model and UTAUT model. Gynecological patients who underwent laparoscopic surgery and met the inclusion and exclusion conditions in a provincial maternal and child health hospital were selected as the research objects. The WeChat intervention group was compared with the nonintervention group, and the oral description score (VRS), comfort score (BCS), and 40-item recovery quality rating scale (QoR-40) were used as the scoring criteria. The results showed that the postoperative VRS and BCS scores in the WeChat intervention group were significantly lower than those in the nonintervention group. The total score of QoR-40 in both groups decreased compared with that before operation, reached the lowest on the first day after operation, and began to rise from the second day. This result is consistent with the patient's postoperative recovery process. After operation, the total score of the WeChat intervention group on days 1 and 2 was higher than that of the non-WeChat intervention group. By comparing the results of the patient's postoperative oral description score (VRS), comfort score (BCS), 40-item recovery quality score scale (QoR-40), etc., it can be shown that the overall recovery quality of the WeChat intervention group was better during these two days. In each section, the oral description score (VRS) and the 40-item recovery quality score scale (QoR-40) indicated that the pain sensation and emotional state scores of patients in the WeChat intervention group were higher than those in the nonintervention group, while the comfort score (BCS) was lower, indicating better comfort in the WeChat intervention group.

## 1. Introduction

With the continuous improvement of medical level, the gradual maturity of laparoscopic technology, and the improvement of mutual learning and communication platform, gynecological laparoscopic surgery is more and more widely used in clinic. Laparoscopic surgery is a newly developed minimally invasive method and an inevitable trend in the development of surgical methods in the future [1]. With the rapid development of industrial manufacturing technology, the integration of related disciplines has laid a firm foundation for the development of new technologies and methods. Coupled with the increasingly skilled operation of doctors, many open operations in the past have been replaced by endovascular surgery, greatly increasing the opportunity of operation selection [2]. The traditional method of laparoscopic surgery is to make three 1 cm small incisions at the patient's waist and insert a pipe like working channel called “trocar” respectively. All operations in the future are carried out through these three pipes. Then the special lengthened surgical instrument is used to complete the same steps as open surgery under TV monitoring to achieve the same surgical effect [3].

Laparoscopy is an endoscope used for intraperitoneal examination and treatment. In fact, it is essentially a fiber light source endoscope, including laparoscopy, energy system, light source system, perfusion system, and imaging system. When applied to surgical patients without pain, it can directly and clearly observe the intraperitoneal situation of patients, understand the pathogenic factors, and perform surgical treatment for abnormal conditions at the same time [4]. Laparoscopic surgery is also known as “keyhole” surgery. Using the laparoscopic system technology, the doctor only needs to open several “key holes” around the surgical site of the patient. Without laparotomy, the doctor can visualize the patient's internal situation in front of the computer screen and perform accurate surgical operation. The operation process takes only a short time, and the treatment technology has reached the international advanced level. The new type of laparoscopic surgery is an operation completed by modern high-tech medical technology with the principle of electronic, optical, and other advanced equipment. It is a cross era progress of traditional laparotomy [5]. It is an operation carried out in a closed abdominal cavity. Under good cold light source illumination, the camera system captures the organs in the abdominal cavity on the monitoring screen through the laparoscopic body connected to the abdominal cavity. Under the monitoring and guidance of high-tech display screen, surgeons operate surgical instruments outside the abdominal cavity for exploration, electrocoagulation, hemostasis, tissue separation, incision, and suturing the diseased tissue [6]. Traditional laparotomy is difficult to operate, with large wound and easy infection. Patients are prone to complications and slow recovery. The new type of laparoscopic surgery is a model of the application of high-tech technologies such as electronics, optics, and photography in clinical surgery [7]. It has the characteristics of less trauma, less complications, safety, and rapid recovery. In recent years, surgical endoscopic surgery has developed rapidly, which can be examined and treated at the same time. It is the most advanced and cutting-edge minimally invasive technology at present.

The concept of rapid postoperative rehabilitation (ERAS) was first proposed by Professor Henrik Kehlet of the University of Copenhagen, Denmark. Its core is to follow the evidence of evidence-based medicine, break the traditional concept, and optimize the clinical treatment and nursing mode during the whole operation period without increasing the readmission rate and reoperation rate [8, 9]. By reducing the traumatic stress response caused by surgery to the human body, this reduces a series of complications that may occur during the whole operation period and finally achieves the purpose of shortening the hospital stay, saving the cost of medical resources, and accelerating the postoperative rehabilitation of patients [10]. After more than 20 years of development, popularization, and application, ERAS concept is more and more widely used in many surgical fields. Its feedback effect is positive, and the results are obvious to all. After ten years of development and application, ERAS has gradually been widely recognized in relevant fields and has formed a series of expert consensuses accepted by most people [11]. However, the concept of ERAS has not been paid enough attention in the field of gynecology, and the available relevant research reports are relatively rare [12]. Since 2014, the application research of ERAS concept in the field of gynecology has gradually increased, involving various surgical methods such as gynecological benign and malignant tumor surgery and uterine prolapse surgery. The application of this concept in the field of gynecology has cross era significance. It shows that people pay more and more attention to gynecological diseases. It also means that we begin to pay more attention to the postoperative recovery effect for the treatment of gynecological diseases, and the postoperative treatment methods of gynecological diseases are more diversified. Nelson et al. summarized and statistically analyzed the literature on the application of ERAS concept in all types of gynecological surgery and ERAS guidelines for abdominal surgery in other disciplines and published a number of guidelines on the use of ERAS concept in the whole operation period in the operation of gynecological benign diseases and gynecological malignant tumors in 2016. The purpose is to provide a unified and standardized standard for the application of ERAS concept in gynecological surgery [13]. ERAS concept guides the nursing mode of postoperative recovery of gynecological diseases, pays more attention to the role of human intervention in nursing, so as to reduce the occurrence of postoperative complications, and advocates standardizing the way of postoperative rapid recovery of gynecological diseases.

Information exchange refers to the communication between individuals with the help of their common symbolic communication system [14]. The “individual” here is generalized and can be an individual, group, or organization. In a broad sense, all activities and processes between information sources and information users belong to the category of “information exchange.” Information exchange is a social phenomenon that has existed since the existence of human society [15]. It is the basic link of information work. With the development of science, technology, and society, the carrier of information, the media, methods, and technology of information exchange are in constant development and change [16]. With the application of modern information technology in the network environment, there are new ways of information exchange, such as e-mail, microblog, WeChat, and so on. Network information exchange is a process in which cognitive subjects exchange and share information with each other by using network technology. Researchers at home and abroad have studied the information exchange behavior of social media from multiple theoretical perspectives, mainly including the network information exchange mode, the conceptual model of the general process of social information exchange, and the integrated technology acceptance theory [17]. This series of theories is suitable for the analysis of the influencing factors of the information exchange behavior of WeChat group users and effectively explains the information exchange behavior of WeChat group users. Chu believes that the application of Wiki is becoming more and more common in different virtual communication. In the research of Wiki, the four elements affecting users' information behavior are community participation, community promotion, community trust, and community identity. Based on the perspective of social network, Liben Nowell studied the prediction of edges in the network and analyzed the structural evolution of the network. Kumar et al. studied the impact of different types of users on the growth environment of social networks [18]. Steinfield and others have studied different social resources in Facebook and found that young users can establish weak contacts outside the circle through their friends. Ellison and others found through the research on SNS website that it can promote users to establish a wider network, and the enthusiasm of users in the network can improve their user capital [19].

This topic aims to explore the intervention role in guiding the rapid rehabilitation after gynecological laparoscopic surgery by means of WeChat.

## 2. Relevant Theories

### 2.1. Unified Model of the First Mock Exam Technology Acceptance and Usage

The unified model of the first mock exam technology acceptance and use is developed by Venkatesh et al. The model is composed of eight different theories of technology acceptance and use: ① reasoning behavior theory; ② technology acceptance model; ③ motivation model; ④ planned behavior theory; ⑤ comprehensive theory of planned behavior and technology acceptance model; ⑥ PC utilization model; ⑦ diffusion of innovation theory; ⑧ social cognition theory. Venkatesh believes that the explanatory power of UTAUT model to users' adoption and prediction is as high as 70%, which is much higher than that of other models. According to UTAUT model, performance expectation, effort expectation, social impact, and promotion conditions are the main factors affecting user adoption [20], as shown in Figure 1.

### 2.2. Information Adoption Model

As for the research on information behavior, most scholars will study a specific link in information behavior, such as user information demand, user information search, and so on [21]. Wilson integrated the specific process of information behavior and proposed a systematic and complete information behavior model. The model completely demonstrated the overall framework from users' information acquisition needs to information utilization for the first time. Since then, most studies on information behavior will refer to this framework for related research [22]. Wilson combined stress coping theory with risk reward theory and social learning theory and proposed a general information behavior model based on the original framework. The new model still takes the user's information needs as the starting point [23]. The difference is that the new model adds five intermediary variables to explore users' information seeking driven by motivation mechanism from the psychological level, demographic level, social level, environmental level, and information source level. The types of information seeking are subdivided into passive attention, passive retrieval, active retrieval, and ongoing retrieval [24]. The model system clearly illustrates the whole process of user information adoption and is suitable for information adoption research. Therefore, this paper selects Wilson's information behavior model as the basic model of WeChat group user information adoption. The establishment of the model makes the adoption process of WeChat official account more clear and convenient for reference, which provides a basis for WeChat to promote the rehabilitation of gynecological laparoscopic surgery.

The specific model diagram is shown in Figure 2:

The specific process of WeChat group user information adoption is as follows: users select health information that meets their own needs by browsing the health information on WeChat group and combining the reliability of health information source and health information content [25]. The specific steps of the information adoption process of health WeChat group users mainly include generating the demand for health information, seeking health information, selection and evaluation of health information, absorption and utilization of health information, etc. Information adoption intention is the premise of information adoption, which will have an impact on the information adoption attitude and behavior of users' health WeChat groups [26]. Based on Wilson's general information behavior model and the characteristics of health WeChat groups, this study proposes the following adoption model, as shown in Figure 3.

Phase I is health information needs. In the trigger stage of information requirements, there are mainly two kinds of information requirements. The first is to clarify the information demand, that is, the unbalanced state formed by the gap between the user's own information state and the user's ideal information state. In order to make up for this unbalanced state, the user will put forward the demand for health information related to the demand. When the user's own health condition has problems, the user tends to know more about the condition. However, in practice, users do not understand it, so an unbalanced state is formed. In this way, when users' emotional cognition is unbalanced (such as the lack of psychological comfort to deal with diseases), they will also seek relevant information. The second is the user's own unconscious health demand, which is the potential health demand; that is, the user browses the health information formed by browsing the circle of friends or being attracted by some forwarded message titles and pictures in the process of reading WeChat group information and browses the health information for adoption. This unconscious health information demand is the potential health information demand. The second stage is health information seeking. Health information seeking includes three steps: information retrieval, information processing, and information integration. The process consists of three parts: information search, information confirmation, and information browsing. In this study, the platform selection section is specifically the health WeChat official account. The third stage is health information selection and evaluation. After searching for information, users will get a large amount of disordered health information. Users must sort out and refine disordered information, so as to quickly screen, identify, and delete the health information that does not meet the demand standards.

## 3. Materials and Methods

### 3.1. Source of the Research Object

The subjects were 250 gynecological patients who underwent laparoscopic surgery and met the inclusion and exclusion conditions in a provincial maternal and child health hospital.

#### 3.1.1. Inclusion Criteria

① Age is <65 years; ② the operative methods were laparoscopic ovarian cyst exfoliation, appendectomy, myomectomy, subtotal hysterectomy, and total hysterectomy; ③ general anesthesia was used; ④ there is no history of intestinal surgery; ⑤ there are no serious internal and surgical diseases; ⑥ there are voluntary collaborators.

#### 3.1.2. Exclusion Criteria

① Those who could not tolerate chewing gum or chewing gum less than 3 times after operation; ② changing the method of eating halfway; ③ intraoperative bleeding often leading to the decrease of Hb to 8/L or below.

#### 3.1.3. Sample Size Estimation

Calculate the sample size and list the formula according to the experimental results.

(1) $$\begin{array}{c} m=\frac{\int_{i=1}^{k}T_{i}^{2}\times \beta_{u1,u2}^{2}\times \left(i-1\right)}{\sum_{i=1}^{k}\left(Y^{2}-Y_{i}^{2}\right)}, \end{array}$$

where *m* is the number of samples required by each group, *K* is the number of treatment groups, and *Y* and *Y*_*i*_ are the estimated values of the mean and standard deviation of the first *i* sample, respectively, which can be found in the table.

Due to the difficulty of manual calculation, the sample size of preexperimental results is estimated by using PASS (Power Analysis and Sample Size) software to calculate the sample size required for formal research.

### 3.2. Intervention Methods

#### 3.2.1. Establishing the WeChat Follow-Up Team

The follow-up personnel are composed of medical staff of hemodialysis center, including 1 deputy chief physician, 1 head nurse, and 5 nurses in charge. All of them have college degree or above, more than 5 years of professional work experience, and good communication, coordination, and expression skills, are proficient in WeChat application, master the operation of various functions, and sign confidentiality agreement. Each of the five nurses in charge is responsible for the WeChat follow-up of 10∼20 patients. After the interview with the patients, a WeChat group is established. In order to protect the privacy of the patients, all patients do not appear with their real names but are included in the group with their nicknames and numbers. The deputy chief physician and head nurse are responsible for formulating WeChat scheme and joining the established WeChat group for communication and feedback and quality supervision.

#### 3.2.2. Establishing the Patient Follow-Up File

Before intervention, WeChat follow-up files were established according to the basic information filled in by patients, and each follow-up information and feedback were recorded in WeChat follow-up files. Team members regularly organized discussion and experience exchange and adjusted and improved WeChat follow-up guidance.

#### 3.2.3. Communication Method

The WeChat group uniformly sends the edited content in the WeChat group, which is generally arranged from 19 : 30 to 20 : 30 in the evening, not during lunch break and night, so as not to disturb the patients. At the same time, it also makes a detailed analysis on the patient's illness and feedback problems and sends the required guidance according to the specific situation of each patient. The transmission frequency is 2∼4 times a week for 1∼3 months and 1∼2 times a week for 4∼6 months, lasting for 6 months. For patients who do not give WeChat feedback in time or show reluctance to participate, understand the reasons, give telephone supervision, and carry out targeted publicity and education, so that they can receive WeChat follow-up education. Pay attention to humanistic care during WeChat follow-up, send WeChat holiday greetings on holidays, remind or invite patients to review time, remind busy people of medication time, etc.

#### 3.2.4. WeChat Follow-Up Content

According to the education level, acceptance ability, and knowledge of kidney diseases of all patients, teach patients the basic knowledge of primary diseases, treatment methods, basic principles of hemodialysis, and various matters needing attention during dialysis. Eliminate patients' anxiety and fear caused by lack of disease knowledge, and carry out targeted psychological guidance according to the situation of patients, help patients establish confidence in treating diseases, and actively cooperate with medical staff in treatment and nursing. Reasonable diet has a great impact on whether to obtain good recovery effect. Therefore, patients must formulate a treatment diet plan in line with their condition and follow this plan in their daily life. In this process, patience is extremely important and should be practiced in person.

### 3.3. Observation Indicators

#### 3.3.1. Verbal Rating Scales (VRS)

It was used to measure the postoperative pain level of all patients. 1 point, painless; 2 points, mild pain, pain does not affect the patient's normal life and sleep; 3 points, moderate pain, pain can affect sleep; patients often require the use of painkillers; 4 points, severe pain, severe pain makes the patient's sleep seriously disturbed, and the autonomic nerve function is abnormal. It is often necessary to maintain a passive posture and take analgesic drugs.

#### 3.3.2. Bruggemann Comfort Scale (BCS)

It is used to evaluate postoperative patient comfort. 0 point, continuous pain in the wound; 1 point, quiet and painless, severe cough, or deep breathing pain; 2 points, lying flat, quiet, and painless, slight pain in cough or deep breathing; 3-minute deep breathing is also painless; 4 points, cough is also painless.

#### 3.3.3. 40-Item Quality of Recovery Score (QoR-40)

QoR-40 scale is an effective measurement tool, which is often used to measure the impact of clinical intervention on postoperative recovery. It has good authenticity, effectiveness, and reactivity. In this study, the scale was mainly used to investigate the early postoperative recovery quality of all patients. The specific methods were as follows: the QoR-40 scores of the two groups before operation and on the 1st, 2^nd^, and 3rd day after operation were recorded through telephone return visit, and then they were simply sorted out and compared.

### 3.4. Statistical Analysis

Establish database with Excel, input patient data, and proofread by two people. The data were statistically processed by SPSS 21.0 software, and the mean and standard deviation were described by quantitative data. The comparison at different time points was analyzed by random block analysis of variance; SNK method was used for pairwise comparison at different time points. *P* < 0.05, the difference was considered to be statistically significant.

## 4. Result Analysis

### 4.1. Total Number of Cases Collected

A total of 958 patients underwent gynecological laparoscopic surgery. In this experiment, 833 cases were finally selected. Among the excluded cases, there were 16 cases with incomplete medical records or inconsistent information with the patients, 7 cases with two or more operations in the same year, and 6 cases with cognitive impairment or mental diseases. 23 cases were complicated with serious systemic diseases, 22 cases were lost to follow-up, and 7 cases died due to invalid contact information or low patient cooperation and inaccurate index information memory. Among the selected patients, there were 422 cases in the WeChat intervention group (W) and 411 cases in the nonintervention group (D), as shown in Figure 4.

### 4.2. VRS Score after Operation

Compared with group W (WeChat Guidance Group), the VRS scores of group D (control group) after operation were significantly lower (*P* < 0.05). The specific results are shown in Figure 5.

According to the research results, the postoperative VRS scores of patients in WeChat intervention group were significantly lower than those in non-WeChat intervention group. It shows that there is a significant difference in the degree of pain between the two groups at different times after operation. The overall analgesic status of WeChat intervention group was better than that of nonintervention group.

### 4.3. Postoperative BCS Score

We also performed BCS scores on 8 groups of patients, and the results are shown in Figure 6. From the figure, we can see that the comfort score of WeChat intervention group is significantly higher than that of the control group. The results show that regular intervention through WeChat group can make patients feel warm, relieve postoperative pain, and accelerate postoperative rehabilitation.

### 4.4. QoR-40 Score

1. There was significant difference in QoR-40 total score of W group at different time points (*P* < 0.001). The total score of QoR-40 in group D was also different at different time points, and the difference was statistically significant (*P* < 0.001). The total score of QoR-40 in both groups increased with the passage of time, as shown in Table 1 and Figure 7.
2. The scores of pain feeling and emotional state in group W were higher than those in group D (*P* < 0.05), and the scores of physical comfort were lower than those in group D (*P* < 0.05). There was no significant difference in the scores of the other parts between the two groups (*P* > 0.05) (Figure 8).

In this study, we evaluated and compared the postoperative QoR-40 scores of the two groups and found that, in general, the total QoR-40 scores of the two groups increased over time. This result is consistent with the patient's postoperative recovery process. After operation, the total score of WeChat intervention group was higher than that of non-WeChat intervention group. It shows that, in these two days, the overall recovery quality of patients in the WeChat intervention group is better. In each part of the score, the pain feeling and emotional state scores of patients in the WeChat intervention group were higher than those in the nonintervention group, while the physical comfort score was lower.

## 5. Conclusion

This study is combined with case analysis to study the intervention role of WeChat group in postoperative rehabilitation of gynecological laparoscopy. In the WeChat group, explain relevant health knowledge and methods to deal with relevant problems to patients, give explanations and psychological help in time, maintain the psychological mood of patients, make them optimistic about life, and improve the oral description score and comfort score of patients.

As a new thing in the field of information technology, WeChat has had a significant impact on the society. Because of its low tariff consumption, high compatibility, and rich information transmission modes, it is favored by more and more people. WeChat follow-up breaks the time and space constraints of medical services. Doctors, patients, and nurses can exchange relevant information through smart phones. The dissemination of information is more accurate, flexible, and personalized. Moreover, the data can be saved in WeChat and is not easy to lose, which meets the requirements of patients' repeated access and learning anytime and anywhere. WeChat intervention plays a certain role in improving the rapid recovery of diseases, and WeChat shows the convenience brought by modern network social tools in the experiment. Different from the traditional intervention methods, WeChat intervention can greatly reduce the cost, avoids the cost of printing leaflets in the past, and also has the advantages of greatly saving time and high attention. In the information age, we need to make full use of the convenience brought by high technology. WeChat has become the best way for people to transmit information. We should also make full use of the advantages of large number of WeChat users, instant sending and receiving messages, not limited by time and place, and saving material consumption, so as to make WeChat compatible with powerful learning functions under the entertainment function. At the same time, new forms of use can also promote the continuous updating of WeChat software and bring more convenient and efficient uses to people. As an intervention means, WeChat platform needs to be constantly updated and improved in its infancy. In the WeChat platform intervention, how to monitor the information sent, how to know whether it has viewed the information, and how to deal with the situation that some intervention objects quit the intervention because they are unwilling to accept the message in the intervention process need to be continuously updated and improved in future research, and better methods should be used to implement the intervention to achieve greater intervention effect.

Although the low WeChat tariff is one of the reasons for its popularity, it is also limited by the Internet in the surrounding environment and the aging of vision with the increase of patients' age. And the knowledge of health educators themselves must be richer and more professional and keep pace with the times, which puts forward new challenges and opportunities for medical workers. In view of the above factors, it is recommended to strengthen the professional management of WeChat follow-up, explore and improve better methods and ways of information arrangement and release, provide patients with higher quality continuous nursing, and effectively improve the quality of life of patients.

## Figures and Tables

**Figure 1:** UTAUT model.

**Figure 2:** Wilson's information behavior model.

**Figure 3:** Information behavior model of the WeChat group.

**Figure 4:** Case collection.

**Figure 5:** Comparison of VRS scores between different groups of patients.

**Figure 6:** Comparison of BCS scores between different groups of patients.

**Figure 7:** QoR-40 score trend of different groups.

**Figure 8:** Postoperative QoR-40 scores.

**Table 1:** Total score of QoR-40.

Group		One month	Two months	Three months	Four months	*P*
First group	W1	176.25 ± 2.71	178.95 ± 4.71	181.33 ± 3.24	187.99 ± 4.23	0.0002
	D1	168.32 ± 5.23	171.29 ± 3.76	174.23 ± 2.87	177.99 ± 6.78	0.0004

Second group	W2	175.36 ± 2.68	179.99 ± 2.23	184.29 ± 5.13	188.49 ± 5.21	0.0008
	D2	165.27 ± 3.44	169.22 ± 4.58	172.44 ± 5.32	176.66 ± 4.18	0.0003

Third group	W3	176.87 ± 4.98	181.22 ± 3.45	188.23 ± 4.48	193.34 ± 5.44	0.0006
	D3	165.25 ± 2.87	168.35 ± 2.55	172.34 ± 3.87	174.22 ± 3.55	0.0009

Fourth group	W4	176.35 ± 3.23	182.55 ± 2355	186.32 ± 4.55	192.35 ± 6.24	0.0001
	D4	168.26 ± 5.68	172.26 ± 4.58	178.46 ± 4.63	182.36 ± 6.56	0.0002

## Data Availability

The data used to support the findings of this study are available from the corresponding author upon request.

## References

[1] Wang T. (2020). Application effect of WeChat group in extended nursing of the patients with indwelling tube after urological surgery during the COVID-19 epidemic. *Advances in Clinical Medicine*.

[2] Huang L., An G., You S., Huang S, Li J (2020). Application of an education model using the WeChat public platform in the standardized training of anesthesiology residents. *Annals of Palliative Medicine*.

[3] Xu Y., Xu L., Zhao W. (2020). Effectiveness of a WeChat combined continuous flash glucose monitoring system on glycemic control in juvenile type 1 diabetes mellitus management: randomized controlled trial,” diabetes, metabolic syndrome and obesity. *Targets and Therapy*.

[4] Chen X., Wu D. H., Xu Z. J. (2019). The effect of WeChat platform in the optimization of emergency treatment for acute ischemic stroke. *Fudan University Journal of Medical Sciences*.

[5] Wu Y., Wall M. (2019). Prosumers in a digital multiverse: an investigation of how WeChat is affecting Chinese citizen journalism. *Global Media and China*.

[6] Qi G., Yi W., Huang Y. (2019). The effectiveness of using a WeChat account to improve exclusive breastfeeding in Huzhu County Qinghai Province, China: protocol for a randomized control trial. *BMC Public Health*.

[7] Phillippi S. W., Luo T., Li M. S. (2021). Urban and rural disparities in a WeChat-based smoking cessation intervention among Chinese smokers. *International Journal of Environmental Research and Public Health*.

[8] Zhen X., Xi W., Zheng L. (2020). One-stage posterior debridement and single-segment interbody fusion for treating mono-segmental lumbar and lumbosacral spinal tuberculosis in adults following minimum 5-year follow-up. *Journal of Orthopaedic Surgery and Research*.

[9] Miao W., Zhang Z., Lu W. (2021). Effect of glucose pretreatment on the effect of rapid rehabilitation surgery in patients undergoing hip replacement. *China Journal of Orthopaedics and Traumatology*.

[10] Vetsheva M. S., Podkorytova O. L., Churakov V. O. (2021). Evolution of approaches in treatment of acute pain syndrome (review). *Medical Alphabet*.

[11] Beekum C. V., Stoffels B., Websky M. V. (2021). Implementierung eines Fast-Track-Programmes. *Chirurg, Der*.

[12] Garmpis N., Dimitroulis D., Garmpi A. (2019). Enhanced recovery after surgery: is it time to change our strategy regarding laparoscopic colectomy?. *In Vivo*.

[13] Tang A., Zhou S. (2021). Analysis on the application value of goal-directed fluid therapy in patients undergoing laparoscopy-assisted radical gastrectomy with fast-track anesthesia. *American Journal of Tourism Research*.

[14] Ioffe O. Y., Stetsenko O. P., Tarasiuk T. V., Kryvopustov M. S. (2019). Perioperative nutrition as an important aspect implementing Fast Track surgery principles. *One Health and Nutrition Problems of Ukraine*.

[15] Romano L. U., Rigoni M., Torri E. (2021). A propensity score-matched analysis to assess the outcomes in pre- and post-fast-track hip and knee elective prosthesis patients. *Journal of Clinical Medicine*.

[16] Wang B. (2020). Therapeutic experience of laparoscopic operation for periappendiceal abscess during the epidemic period of novel coronavirus pneumonia: a case report. *Hans Journal of Surgery*.

[17] To A., Tanaka B. N., Oyama C. A. (2020). fficacy and safety of low-molecular-weight heparin on prevention of venous thromboembolism after laparoscopic operation for gastrointestinal malignancy in Japanese patients: a multicenter, open-label, prospective, randomized controlled trial – ScienceDire. *Journal of the American College of Surgeons*.

[18] Feng X., Cao J. S, Chen M. Y (2020). Laparoscopic surgery for early gallbladder carcinoma: a systematic review and meta-analysis. *World Journal of Clinical Cases*.

[19] Hideki (2019). “[Palliative laparoscopic operation for an extremely elderly patient with cecum cancer],” Gan to kagaku ryoho. *Cancer & chemotherapy*.

[20] Ramsay G., Scott N. W., Jansen J. O. (2020). A 19 year population-based cohort study analysing reoperation for recurrence following laparoscopic and open inguinal hernia repairs. *Hernia: The Journal of Hernias and Abdominal wall Surgery*.

[21] Yang M., Wen S., Huang Y., Hua Y. (2020). The effect of laparoscopic two-staged Fowler-Stephens operation on prognosis in children with high intra-abdominal testicles: an observational study. *Asian Journal of Surgery*.

[22] Ling K. J., Wang Y. Z., Zhang H. (2021). Oncologic outcomes of early stage cervical cancer performed operation by different laparoscopic surgical procedures: analysis of clinical data from mutiple centers. *Zhonghua Fu Chan Ke Za Zhi*.

[23] Biyik İ., Albayrak M., Keski̇n F., Mut A. N. (2020). The effect of uterine manipulator use in laparoscopic tubal ligation on operation duration and anesthesia drug quantity. *Journal of Clinical Obstetrics & Gynecology*.

[24] Feleshtynskyi Y. P., Shtaier A. A. (2021). Morphological justification of laparoscopic transabdominal preperitoneal (TAPP) operation for the inguinal hernia recurrence. *Journal of Education, Health and Sport*.

[25] Khaled I., Abouali M., Gomaa M., Eldeeb A. E., Gabr H., Soliman A. (2020). Evaluating the efficacy of laparoscopic mini-gastric bypass operation in reducing weight among obese patients. *Suez Canal University Medical Journal*.

[26] Yüce D., Salman S., Kumbasar S., Tuna G. (2020). Strangulated small-bowel loop herniation at the 5 mm trocar entry site after laparoscopic ovarian cyst excision operation. *The New Indian Journal of OBGYN*.

